# Design of Mobile English Teaching Platform Based on Collaborative Filtering Algorithm

**DOI:** 10.1155/2022/7566896

**Published:** 2022-07-31

**Authors:** Cong Xu

**Affiliations:** School of Foreign Languages, Hubei University of Science and Technology, Xianning 437100, Hubei, China

## Abstract

With the rapid development of information technology, today's talent training mode is no longer limited to traditional school education. At the same time, with the maturity of portable mobile devices, a new learning method—mobile learning has been born. In this paper, the narrative of data is taken into account in the way of user collaborative filtering recommendation. For prefilling the matrix, the project confidence level also needs to be considered during the whole process. The project confidence level is measured by information entropy model. In the process of correction, it combines with traditional cosine similarity, calculates the user similarity matrix, can budget equalization, and expands the original matrix. After filling the matrix, the user uses the method of similarity calculation, using Pearson similarity and combining with the Euclidean distance correction method. When comparing the particular result prediction with the actual prediction following the completion of the similarity matrix data, all results point to a considerable reduction in MAE and RMSE. The user does not assess the item score to forecast. This demonstrates how this technique may enhance the reliability and consistency of the mobile English system platform.

## 1. Introduction

With the advent of modern era especially in the field of communication and technology has enabled people across the world, irrespective of how long the distance is between them, to communicate with each other preferably with minimum possible cost or overhead. Additionally, these devices are very common and within the feasible range of the ordinary human being. As the technology grows, communication protocols and ways are also improved with the passage of time to make these consistent with the advance devices which are introduced with the passage of time. Nowadays, we can communicate via these electronic devices with other parties that reside in every corner of the world using either audio or video or both communication mechanisms. In addition to the communication, these devices or networks could be an alternative way or means of online teaching, i.e., distance learning, which are programs introduced by various universities to ensure door-to-door education where applicable.

Now there are more and more Internet users around the world. China's Internet users already account for 20% of the total number of people in the country. They are also one of the top 10 Internet giants in the world. They have a strong network power. At home, they have been continuously strengthening the network technology, and take the scientific development as the basis for active use. With the continuous formation and deployment of the mobile network by 4G network, the transmission speed is faster and faster, which has greatly promoted the development of the Internet and has reached its peak. The whole country has gradually started to implement 5G technology. In the process of commercial development, the low delay and high speed of 5G network has played a great role and has become an irreplaceable technology. Mobile Internet has now been able to form a fast combination of online and offline. Combining the two methods in traditional industries, the industries can find a broader space for development. The development of society cannot be separated from the support of education, and the mobile Internet has also brought greater reform to the education industry [1].

Utilizing personalized recommendations can help solve this type of problem, which is also very helpful for the development of education platforms. At this stage, collaborative filtering recommendation algorithm has the greatest advantage over other traditional algorithms for personalized recommendation, which is very practical for unstructured online learning resources. By using this strategy to mine prospective user signals in the case of low user ratings in MOOCs, for instance, the accuracy of push may be ensured [2].

The main contributions of this paper are as follows: (1) collaborative filtering recommendation develops rapidly with its advantages, focusing on the relationship between the project and users, rather than considering the specific content between users and projects, so the whole process has strong adaptability, and can form personalized recommendation and intentional recommendation. (2) The method used in this paper is based on collaborative filtering of personality recommendation and has been widely used in online education platform. (3) Based on the theory of information entropy, this paper puts forward projects with different confidence, and the number of evaluations used is also different. User interest is also shown by the higher number of evaluations, which means that users have a higher degree of interest. User interest is measured by the degree of project execution.

Organization of the remaining article is given below.

Related work is presented in the section just following where historical studies related to the problem domain are reported and described how the issues can be solved by using these techniques. Next in Section 3, improvement of similarity calculation method for collaborative filtering is reported which is actually the technique proposed in this article. For easy follow-up, this discussion is divided and presented in separate sub-sections of the paper. In Section 4, design of mobile English teaching platform based on collaborative filtering algorithm is reported and how this model is a solution for the problem at hand is described in an easy-to-follow way. Various simulation results which are observed during the experimental setup, i.e., simulation setup, are presented in both form that is graphical and textual. Lastly, summary of the proposed and existing work along with references is reported in the conclusion section.

## 2. Related Work

At the end of the last century, Tapestry pointed out that it was the basic recommendation system model, and more and more scholars have paid attention to it and continuously improved it. This has been one of the hot topics and is growing rapidly [3]. There are four main types of methods used by different websites or systems: content-based recommendation, collaborative filtering, association rules, and mixed recommendation. Collaborative filtering has been used in many areas because of its many advantages and good performance, and more and more organizations and scholars focus on it [4–7]. In the essay, Goldberg introduced the synergy probability and demonstrated Tapestry's filtering for the first time. You must enter your individual demands in the search field to find previously read articles using a rating technique. Based on the user's search information, you can then suggest comparable remarks [8]. An automated-like collaborative filtering technique was put out by Cheema et al., investigating and assessing past consumers' choices for network news was the key focus. Assuming that users' tastes would not significantly alter in the near future, we may create later-stage user preferences, anticipate models, and offer suggestions for more intriguing news [9]. After new users join, not too many news reviews can be used to view users with similar interests or to recommend those who have recently browsed similar news [10]. This method can be more in line with users' preferences. Conducting a specific analysis of news content can not only recommend content to users' preferences, but also improve performance. This recommended approach is now used in many areas [11].

Considering the increasing data growth of projects and users, collaborative filtering has certain restrictions on balancing data scarcity and its limitations. Mao and Tang used information theory to measure and evaluate the relevance of features, which can ensure the weighting of features or the selection of items. They can continuously improve the way of learning synchronization and ensure the accuracy and efficiency of recommendations [12]. The collaborative filtering method proposed by Zhang et al. is based on user time weights, which can better solve [13] the startup problems of current projects. Wang et al. adopted copper wash filter, the recommended algorithm is based on the uncertain forest entry method, mainly for the adaptive prediction method used in unpredictable situations, and for the near target selection [14]. The traditional collaborative filtering algorithm used in the recommendation process must be mastered for the user's rating information, but in the actual process, there is very little rating data. If some new users are lazy, they will not rate the commodities. This will not guarantee the quality of recommendation. In order to improve the accuracy of prediction, Mining for user-rated information is the main direction [15]. The collaborative filtering method proposed by Wang et al. is based on the cloud model, which is used to calculate the similarity between users in the case of sparse data, so as to ensure the accuracy of system recommendations [16].

## 3. Improvement of Similarity Calculation Method for Collaborative Filtering

Similarity of data value plays a vital task in the development of a precise and accurate filtering scheme, i.e., the one proposed in this section. In literature, various approaches are available for the computation of similarity indexes between two or more datasets, however, each mechanism has certain advantages and disadvantages, i.e., these algorithm may work outstanding in certain scenarios, but may not be good for other data sets.

### 3.1. Defects of Traditional Similarity Calculation Method

#### 3.1.1. Scoring Criteria Question

For the traditional collaborative filtering calculation method, the result is that the cosine similarity can be corrected, or for the scoring standards between users, it needs to be measured by a comprehensive consideration, using the method of subtracting the average score, expanding the corresponding constraints, considering the absorbability of data, and measuring the standards between two users. Users can receive information that they are interested in, and almost all that another users receive information that they are not interested in. As shown in Table 1, all *u*_1_ users score less than or equal to 3 points, indicating that they are not interested and that all *u*_2_ users score more than 3 points, indicating great fun, although the average score is subtracted from the algorithm. However, the similarity of *sim*(*u*_1_, *u*_2_)=1 is unreasonable and needs to be continuously improved.

#### 3.1.2. Share of Common Scoring Items

When calculating similarity between users, traditional joint filtering calculation methods usually find elements that two users evaluate at the same time to calculate the similarity of the estimates. However, due to the scarcity of data, only a few assessable elements in the rating matrix are used by different users, resulting in very high similarity, although there are few general rating elements. Therefore, when selecting the nearest K-neighbor among the user group, few people who have common evaluation elements participate in the unknown prediction evaluation due to high similarity, which will greatly reduce the accuracy of the system. As shown in Table 2, 0 represents no estimate, the common estimate elements for *u*_1_ and *u*_2_ users are only *I*_1_, the same estimate, and the similarity value is 1. Common elements of *u*_1_ and *u*_3_ user evaluations are *I*_1_, *I*_2_, and *I*_4_. Due to the different estimates of *I*_1_, the similarity is lower than *u*_1_ and *u*_2_, which is also an inappropriate value.

### 3.2. Improvement of Similarity Calculation Method

#### 3.2.1. Improvement Method

It is important to note that it would be considered as a plus if we could possibly improve the performance of the similarity computation method, i.e., existing one, without compromising on other evaluation metrics. Some of these improvement mechanisms are described below in detail.

(1) Penalty mechanism for scoring criteria: from the above analysis, it can be known that when analyzing the user's rating criteria, the problem that the average value of all user's rating needs to be subtracted from that of the rating criteria has been better solved. However, the data used is a randomly extracted part of the users and the corresponding rating is made for some interesting or uninteresting items, so the result is not accurate or low. There may also be a high degree of similarity between the two users, which does not match the actual situation, and inaccuracies may occur during the recommendation process [17]. This subsection gives the difference between two users of the same item, as shown in the following formula:
  (1) $$\begin{array}{c} d=\frac{r_{u,j}-r_{v,j}}{N}. \end{array}$$
  Here, *r*_*u*,*j*_ and *r*_*v*,*j*_ represent *u* and *v* user ratings under *j*, respectively. The maximum allowable rating for the system is *N* and the maximum rating in this chapter is 5. The difference between the score of the same *u* user and *v* user and the highest score supported by the system is a good measure of the difference. Restrict the users who have different average scores and similar deviations in order to measure their similarity more accurately.
(2) Mechanism for penalizing items with low common scores: some users will contribute less because of the lower common rating items indicated in the prior article. The proportion is likewise rather high when predicting the scoring. Overall, user interest is mostly reflected in the common average score. Users often select the sort of English workouts they are interested in finding without considering any other aspects. Different users have a great degree of intersection with different types of English practice systems. In a certain direction, the two users may have the same interest, so the similarity between the two users is relatively high, which can be measured by means of a common equalization or expressed by Tanimoto coefficient [18]. Based on the following formula the common score item proportion is utilised for the intersection of users in order to increase similarity or prevent lower item scoring among users.
  (2) $$\begin{array}{c} T\left(u,v\right)=\frac{\sum \left(u_{i}\cap v_{i}\right)}{\sum \left(u_{i}\cup v_{i}\right)}. \end{array}$$

#### 3.2.2. Construct Similarity Measure Formula

Similarity between users can be influenced by different rating standards or by lower common rating items, and various solutions are presented above. This section modifies the Tanimoto coefficient by combining the fractional difference between different users with the Tanimoto coefficient.

(3) $$\begin{array}{c} {\text{sim}}_{2}=\sum \frac{\left(u\cap v\right)-\left(u\cap v\right){\left(r_{u,j}-r_{v,j}/N\right)}^{2}}{\left(u\cup v\right)}. \end{array}$$

As shown in formula (3), the smaller the *r*_*u*,*j*_ − *r*_*v*,*j*_ value, the smaller the fractional difference, (*r*_*u*,*j*_ − *r*_*v*,*j*_/*N*)^2^ fractional difference. When *u* > v is larger, it means there are more general evaluation elements. In both cases, the value *u*∩*v*(*r*_*u*,*j*_ − *r*_*v*,*j*_/*N*)^2^ is small, and the modified Tanimoto can better hide large score differences between users and less common problems with score elements, ensuring the accuracy of calculation.

In the process of recalculating the user similarity matrix, it is necessary to combine the traditional related similarity formula with the modified Tanimoto coefficient, as indicated by the following formula. The final calculation method used is SIM.

(4) $$\begin{array}{c} {\text{SIM}=\text{sim}}_{\text{pcc}}+{\text{sim}}_{2}\text{.} \end{array}$$

## 4. Design of Mobile English Teaching Platform Based on Collaborative Filtering Algorithm

Teaching is one the most valuable and trustable profession in the world and every teacher tries his best to deliver his/her knowledge to the student in an effective and easy-to-follow ways. However, teaching style and methodology of every teacher is different which makes it difficult for certain class of student to follow it. Moreover, with the advent of modern technology, teaching platform could be more useful if technology is adopted, then not only it could be more useful for the teacher as lecture delivery will become easier, but at the same time, it could be more beneficial for students as they can record lectures and can listen to it repeatedly, if they did not understand a topic at the first go. Secondly, it could be a positive point for those student who misses a class due to some reasons. Some of the filtering mechanism are described below.

### 4.1. Filling Algorithm Based on Item Confidence

Confidence Level of Projects: the orderliness of the information theory system as a whole is mentioned above, and information entropy is used to represent the degree of project execution in this chapter. In the process of system validation for users and the number of projects, it is found that the problem of increasing system scarcity will certainly occur. If a user scored less for a project and then calculated its similarity, the overall calculation may be somewhat contingent [19, 20]. Few individuals have given the project much attention, and just a few have given it a score, indicating that the project has little interest and that it is hard to discern whether it is being measured. It will thus have more unpredictability or chance if fewer people pay attention to it, which is why this chapter introduces the project confidence research.

In Table 3, when the similarity between user *u*_1_ and *u*_3_ is calculated, only *I*_1_ and *I*_2_ are scored together. *I*_2_ is too low for all users to be universally scored. In this case, the same score on *I*_2_ will increase the similarity between user *u*_1_ and *u*_3_, thus making the calculation inaccurate. This chapter introduces how information entropy defines the confidence level of an item, and the probability of *I*_*x*_ appearing is shown in the following formula:

(5) $$\begin{array}{c} p\left(I_{x}\right)=\frac{\text{count}\left(I_{x}\right)}{\text{count\_user}}. \end{array}$$

In the above formula, count(*I*_*x*_) is the number of times that item *x* is evaluated, count_user represents the total number of users, and then defines the information entropy of *I*_*x*_. Items with higher information entropy have greater confidence, discrimination, and contribution to the calculation of similarity. As shown in the following formula, *H*(*I*_*x*_) represents information entropy.

(6) $$\begin{array}{c} H\left(I_{x}\right)=-p\left(I_{x}\right)\log\;p\left(I_{x}\right). \end{array}$$

The traditional cosine similarity calculation method mentioned above is shown in the following formula:

(7) $$\begin{array}{c} {\text{sim}}_{3}=\frac{\sum \left(r_{u,j}\times r_{v,j}\right)}{\sqrt{\sum {\left(r_{u,j}\right)}^{2}}\times \sqrt{\sum {\left(r_{v,j}\right)}^{2}}}, \end{array}$$

where *r*_*u*,*j*_ and *r*_*v*,*j*_ represent user *u* and *v*'s rating of project *j*, respectively.

Corrected cosine similarity with weighted item confidence is shown in the following formula:

(8) $$\begin{array}{c} {\text{sim}}_{4}=\frac{\sum \left(r_{u,j}\times H\left(I_{x}\right)\times r_{v,j}\times H\left(I_{x}\right)\right)}{\sqrt{\sum {\left(r_{u,j}\times H\left(I_{x}\right)\right)}^{2}}\times \sqrt{\sum {\left(r_{v,j}\times H\left(I_{x}\right)\right)}^{2}}}. \end{array}$$

Here, *H*(*I*_*x*_) is the information entropy of item *x* and *r*_*u*,*j*_ and *r*_*v*,*j*_ have the same meaning. The improved formula calculates the similarity matrix between different users and finds each user's nearest neighbor to fill in items that the user has not rated.

Based on the user similarity matrix calculated above, the user unrated item score can be obtained from the following formula, which prepopulates the original matrix.

(9) $$\begin{array}{c} P_{u,j}=\frac{\sum {}_{v∍k\left(u\right)}{\text{sim}}_{4}\left(u,v\right)\times r_{v,j}}{\sum {}_{v∍k\left(u\right)}|{\text{sim}}_{4}\left(u,v\right)}. \end{array}$$

Here, *P*_*u*,*j*_ is the final predictive score for the item, *k*(*u*) is the nearest neighbor set, sim(*u*, *j*) is the similarity factor, and *r*_*u*,*j*_ is the user *v*′s score for item *j* in the nearest neighbor set.

### 4.2. Server-Side Construction of Mobile Learning System

An online platform for education that is built on SSH serves as the server for the mobile learning system. For deployment, the data accepts SQL Server 2008 and Mono, and transits over Apache Tomcat 8.

1. A distributed deployment scheme based on MongoDB and SQL Server databases: as the number of users in the mobile learning system increases, data requests increase at the same time, and the load on the database increases. Based on this consideration, and combined with MongoDB data replication and fragmentation mechanism, a distributed data processing mechanism based on MongoDB and SQL Server is designed. Through SQL Server, the teaching tasks assigned by teachers on the network platform on September 1 are managed, and based on MongoDB, data operations frequently requested by students, such as homework, examination sending, status saving and change, are handled.  Figure 1 shows the interaction with the mobile learning system.
2. The server-side database of the mobile English system uses the combination of SQL Server + MongoDB and is developed in MVC mode. Data is returned to the client in JSON data format and distributed clusters are used to solve a large number of simultaneous client access problems. The server structure is shown in Figure 2.

## 5. Analysis of Experimental Results

In this section, a detailed analysis of various results, which are observed during the simulation setup while comparing performance of the existing and proposed work, are reported here one by one.

### 5.1. Analysis of Similarity Calculation Results

According to the MovieLens open source data set, 80% are randomly selected for learning and 20% for testing. The improved algorithm is used to predict the missing 20% data and compared with the data in the test set. The root mean square error is calculated to measure the prediction accuracy. According to the difference of nearest neighbor value *K*, the traditional joint filtering algorithm is compared with the improved joint filtering algorithm in this paper.

The estimated index data obtained after experiments with traditional cooperative filtering methods and improved algorithms are shown in Figure 3.

As seen in Figure 3, the methods in this chapter are compared to Tanimoto similarity, cosine similarity, and Pierson similarity in the conventional aggregate filtering technique. The algorithm in this chapter is more accurate than the conventional similarity algorithm. When compared to the conventional analogy technique, the algorithm in this chapter has an average Mae of roughly 8% if *K* is equal to 10. In order to lessen the detrimental effects of uncommon data, when *k* is equal to 20, it has strong stability and may produce more accurate prediction results without requiring additional neighboring sets.

As shown in Figure 4, this figure compares the valley similarity, cosine similarity, and correlation similarity in the traditional joint filtering algorithm with the root mean square error difference of the algorithm in this paper under different nearest neighbors. It can be seen from the figure that the RMSE value of the algorithm in this paper is the best, which is higher than that of the traditional algorithm. When the value of *K* is 10, the root mean square deviation of the algorithm in this paper is about 7.3% lower than that of the traditional similar algorithm. When the value of *K* is 20, it also tends to converge. If the data is sparse and the number of nearest neighbors is small, the algorithm in this paper can also predict the best result of accurate data with small deviation from the original data.

### 5.2. Result Analysis of Improved Collaborative Filtering Algorithm

In this paper, a new similarity measurement method is constructed by the formula, the similarity between different users is calculated, and then the similarity neighborhood of the target user is obtained. After the similarity decreases, the first *k* nearest neighbors, that is, the similarity neighborhood of the target user, are selected. The estimated value of the element is predicted according to the estimated value of the element closest to *K* and suggestions are generated.

According to the MovieLens open source data set, 20% are chosen at random for testing and 80% are chosen at random for learning. The data in the test set are compared with predictions made using the improved algorithm for the 20% of the data that is missing. To determine the accuracy of the forecast, the root mean square error is determined. The standard joint filtering technique and the upgraded approach are contrasted in this research based on the difference in *K* value. Figures 5 and 6 demonstrate this.

As shown in Figures 5 and 6, the traditional joint filtering algorithm is compared with the algorithm described in this paper. It can be seen from the figure that the accuracy of the algorithm in this paper is higher than that of the traditional similar algorithm. When the value of *K* is 10, the average Mae of the proposed algorithm is reduced by about 7%, and the average RMSE is reduced by about 6% compared with the traditional similar algorithm. When *k* is 20, it tends to converge, so it has good stability. More accurate prediction results can be obtained without providing more neighborhood sets.

### 5.3. Performance Test Results of Mobile English System

This paper uses Baidu mobile cloud test center and Testin cloud test automation test platform to download the APK and test cases of mobile learning system to the platform. MTC test platform accepts the test of 20 top mobile phones in the market and selects them on the Testin cloud test platform. 100 mobile phones are basically tested, and 100 mobile phones are divided into 4 groups. The average stability rate and compatibility ratio of the above four groups of tested mobile phones are calculated. After the platform automation test, receive the software test report is received. The test results are shown in Table 4.

From the analysis of the above test results, it can be seen that some mobile phone system compatibility problems were found in the test process of the new mobile phone of top-20 on MTC test platform and 100 mobile phones on Testin test platform. Some mobile phones are matched with software, and some mobile phones have insufficient compatibility.

## 6. Conclusion

This paper focuses on the process of the algorithm and the improvement of related problems, makes a detailed analysis of the theoretical part, improves some shortcomings of the traditional collaborative filtering algorithm, and puts forward the scoring standard punishment mechanism and the low common scoring item punishment mechanism. The experiment demonstrates that the modified method has significantly improved Mae and RMSE values under the same conditions and can also provide decent results when the data is sparse, considerably addressing the drawbacks of the conventional recommendation system. The experiment demonstrates that the enhancement enhances the algorithm's performance. The theoretical portion mentioned above is implemented in the mobile English system platform by utilizing the system technique and concentrating on the English recommendation system subsystem for the previously mentioned enhanced algorithm. The algorithm produces improved recommendations for various users.

## Figures and Tables

**Figure 1:** Fragmented database connection.

**Figure 2:** Server architecture.

**Figure 3:** Mae corresponding results under different recommended methods.

**Figure 4:** RMSE corresponding results under different recommended methods.

**Figure 5:** Mae corresponding to different similarity measurement methods.

**Figure 6:** RMSE corresponding to different similarity measurement methods.

**Table 1:** User rating criteria matrix.

	*I*_1_	*I*_2_	*I*_3_	*I*_4_
*u*_1_	3	2	3	2
*u*_2_	6	5	6	5

**Table 2:** User shared rating matrix.

	*I*_1_	*I*_2_	*I*_3_	*I*_4_
*u*_1_	5	2	0	4
*u*_2_	3	0	1	0
*u*_3_	4	0	1	3

**Table 3:** User rating matrix.

	*I*_1_	*I*_2_	*I*_3_	*I*_4_
*u*_1_	5	1	0	3
*u*_2_	5	0	1	0
*u*_3_	2	0	0	3
*u*_4_	5	1	1	4
*u*_5_	1	0	2	3

**Table 4:** Systematic test results of mobile English on 100 experimental mobile phones.

Test group	Average stability rate (%)	Compatible proportion (%)
Group 1	90.2	90.5
Group 2	91.5	89.8
Group 3	89.6	85.5
Group 4	92.4	90.4

## Data Availability

Data are available on request from the corresponding author.
